# Segmentation and Classification of White Blood Cells Using the UNet

**DOI:** 10.1155/2022/5913905

**Published:** 2022-07-11

**Authors:** Amal H. Alharbi, C. V. Aravinda, Meng Lin, P. S. Venugopala, Phalgunendra Reddicherla, Mohd Asif Shah

**Affiliations:** ^1^Department of Computer Sciences, College of Computer and Information Sciences, Princess Nourah bint Abdulrahman University, P.O. Box 84428, Riyadh 11671, Saudi Arabia; ^2^N. M. A. M Institute of Technology Nitte, Karkala, India; ^3^Department of Electronics and Computer Engineering, College of Science and Engineering, Ritsumeikan University, Kyoto 525-8577, Japan; ^4^University of Central Missouri, 116 W South St, Warrensburg, MO 64093, USA; ^5^Bakhtar University, Kabul, Afghanistan

## Abstract

In the bone marrow, plasma cells are made up of B lymphocytes and are a type of WBC. These plasma cells produce antibodies that help to keep bacteria and viruses at bay, thus preventing inflammation. This presents a major challenge for segmenting blood cells, since numerous image processing methods are used before segmentation to enhance image quality. White blood cells can be analyzed by a pathologist with the aid of computer software to identify blood diseases accurately and early. This study proposes a novel model that uses the ResNet and UNet networks to extract features and then segments leukocytes from blood samples. Based on the experimental results, this model appears to perform well, which suggests it is an appropriate tool for the analysis of hematology data. By evaluating the model using three datasets consisting of three different types of WBC, a cross-validation technique was applied to assess it based on the publicly available dataset. The overall segmentation accuracy of the proposed model was around 96%, which proved that the model was better than previous approaches, such as DeepLabV3+ and ResNet-50.

## 1. Introduction

The disorders in the blood cells are diagnosed in the laboratory using blood microscopy. The accuracy of the results depends on the pathologist/hematologist. Leukocytes, RBCS, and platelets are the three main components of blood. Doctors will be able to identify blood diseases such as blood cancer, anemia, and malaria using micrographs recorded using computer-aided techniques. An important feature of white blood cells is the type and count of leukocytes, which determine the type and severity of infection. WBCs that are having small granules are further categorized as neutrophils, basophils, and eosinophils. There are three types of leukocytes that make up the immune system. The traditional method of counting white blood cells is laborious and requires medical expertise. Cell segmentation and feature extraction are required for the analysis of WBC. In the process of white blood cell segmentation, leukocytes are extracted from blood smear images to find the necessary features for further processing to distinguish them from others. There are two types of segmentation techniques: boundary-based and region-based. In image processing, segmentation helps to identify the objects in an image. Region-based techniques segment images use properties like those of boundaries; boundary-based techniques and segmented images are based on changes in intensity at the boundary. To distinguish WBC from the background, we applied the region-based segmentation. Due to the irregularity of the shape of leukocytes, it is a challenging task for the segmentation process. For example, Figures 1 and 2 show various types of white blood cells along with their ground truth images. Literature indicates that few automated systems are presently available to analyze blood smear images for leukocytes. Research is in progress to design a system that automatically segments leukocytes with maximum accuracy in a short amount of time. In some studies, the authors use algorithms to segment merely WBC, while in others, they also publish methods for segmenting the nucleus and the cytoplasm [2, 3].

The two parts of WBC are the unsupervised learning model and supervised learning model. Thresholding [4, 5], clustering-based technique [6], fringe-situated [7], zone-positioned [8], and fuzzy models [9, 10] are used in unsupervised learning. Based on the supervised algorithm, every pixel was categorized into two in the ROI and nonregion of interest. To enhance detection, DLN was used in segmenting the images. DLN was found to be a useful concept in medical image analysis due to its performance. Deep learning-based models require a large amount of memory and processing resources for training and testing data. The system is trained repeatedly faster on GPUs than on CPUs [11]. Deep learning-based segmentation consists of instance segmentation and semantic segmentation. During instance-based segmentation, the mask is used to detach different ROIS and utilizes masks to classify the images. To characterize WBCs as shown in Figure 3, based on the mononuclear cells, it can be divided into either mononuclear or polynuclear cells [12]. The thresholding method has been used in several prior studies to analyze blood cell frequency to detect cancer. However, finding the optimal threshold value is laborious and complex; nevertheless, previous studies have used this methodology for cancer detection. CNN models can extract thousands of features from images automatically; therefore, we used it, and so, they can extract thousands of features from images automatically. It takes a long time to manually extract many features, whereas CNN models can extract thousands of features quickly and accurately. The segmentation of leukocytes was accomplished using the more accurate model developed to determine the boundaries of internal cells at the cellular level. This implementation can transfer information from encoder to decoder with no loss of detail while avoiding losing the microdetails. The focus of this research is to build a system that can accomplish the task of segmenting and classifying WBC, enabling physicians to easily determine the exact position of a myeloma cancer cell.

## 2. Literature Review

This section covers the research articles of various researchers who worked on the method of detecting cancer cells in WBCs by using an image processing algorithm to detect myeloma, which is developed as discussed in [13]. A research article by Joshi et al. covered the portion to classify and segment WBC for the diagnosis of leukemia. They applied the Otsu algorithm to enhance and segment WBC. The K-nearest neighbors (KNN) classifier has been used to identify myeloma from normal B cells [14]. Liu et al. worked towards classifying and recognizing using the ML algorithm to extract data. Artificial intelligence utilizes image recognition technology. Intelligence is based on the concept of analyzing data using digital images that can be processed using a computer and then extracting data from them [15]. Martinez et al. illustrated low-dose CT images for detecting myeloma in the bone marrow [16]. Xu et al. worked on image classification as well as the type and position of objects [17], VGG [18], inception [19], fuzzy logic [20], Faster R-CNN [21], SSD [19], and YOLO [11], which are all methods for segmentation and object detection. They concluded that for image classification, they had been using a statistical deep learning framework that emphasized object categorization inside the image [22, 23]. DL segmentation is broadly classified into instance and semantic segmentation, identical masks are used for ROI, and semantic is used for a single image. This approach recognizes individual cells instead of classifying four cells as one instance. The proposed research work will be carried out on semantic segmentation using the CNN to segment WBC cells.

From the above literature, it is found that the existing models suffer from hyperparameters tuning [1, 24–26], gradient vanishing [27, 28], and overfitting [29–31] problems. Therefore, an efficient model is required that can overcome these issues.

## 3. Resources and Methods

ISBI C-NMC 2019 data were used in this study. Approximately sixty cancer patients' datasets were collected and forty-one individuals were added to this dataset. In total, around ten thousand six hundred cells are with a train, validation, and test split of 80%, 10%, and 10%, respectively [12]. To maintain integrity, the first steps of preprocessing are standardization and normalization. These images were first calculated to find the global mean and standard deviation (STD). The following equation is normalized equation , where $\bar{y}$ indicates the global mean Yi of the image equation, the STD, and *ε*=le − 10. The training dataset underwent data augmentation.

(1) $$\begin{array}{c} \text{Yi}=\frac{\text{Yi}-\bar{Y}}{\sigma +\varepsilon }. \end{array}$$

WBC segmentation is carried out using the MASK-RCNN network for blood images through the semantic segmentation process; meanwhile, these WBCs relate to positive classes and their pixel relates to negative, which is shown in Figure 4; for the input images, the initial process to train the model, ResNet [1, 24] was scaled to 224 ∗ 224 to maintain stability and to scale the output of the network. Later, for the ground truth, sample labels were applied to each pixel by making them to the chosen label/class. A variety of convolutional algorithms [25, 26] followed by postprocessing techniques were applied to enhance future extraction for classification [27, 28] during the decoder phase.

### 3.1. Process of Semantic Segmentation

This is a type of pixel-level image classification; during the segmentation process, every pixel present in the image will be categorized into one predetermined group. In the blood sample, there will be several leukocytes; while doing segmentation, each WBC pixel will be labeled as an object, such that it will help in the recognition and classification of leukocyte types present in the sample. However, during feature extraction through the deep layer network, due to large layers, this will lead to gradient descent. To overcome these issues, the ResNet model was used, the advantage of using this model was to prevent the colloidal occurring in the layers and combine their outputs. To calculate the loss that was the expected value and the gained value, the backpropagation algorithm technique was implicated. The complexity of this technique will consume a large amount of memory. To solve these issues, the encoder and decoder were combined for upsampling and downsampling. The traditional CNN algorithm [29, 30] will calculate the probability for each class label, but upsampling will change the output dimensions in such a way that matches the input dimensions. This proposed architecture for segmentation tasks has several advantages. To start with, residual units assist in deep learning. A second advantage of accumulating features with recurrent residual convolutional layers is that they enable better feature representation. Third, it enables us to design better UNet [31] architecture with the same number of network parameters, while obtaining better performance for medical image segmentation.

### 3.2. UNet Architecture

In this architecture, there are three main features, namely, feature reconstruction, feature extraction, and feature fusion. During the process of feature extraction, the location-based feature encoder was mainly used to extract multiscale features based on convolutional blocks and residual blocks.  Figure 5 shows that to modify the feature maps of the given image size, convolutional and deconvolutional techniques were applied to the sample for reconstructing the feature stage. The developing and expansive paths consist of three layers in each path of blocks, where each layer will follow 2 ∗ 2 max pooling on the developing path. In the convolution process, the two layers of upsampling are concatenated with the two layers of merging layers. To generate the pixel-by-pixel value scores, a 1 ∗ 1 layer was activated with the sigmoid function to be used as the final output layer. In every layer of the block like 1, 2, and 3, the layer consists of 112, 224, and 448 filters, whereas the expansive path consists of 224, 122, and 122, respectively. Original UNet architecture and proposed CNN dropouts were used on the expansive path, as given in Table 1.

### 3.3. Layers of the Proposed Model

The layers of the proposed model used are given in Table 1.

### 3.4. Process of the ResNet Architecture Model

This model consists of 50 layers, and CNN blocks were being used several times in this architecture. In every layer, it consists of a batch normalization of 2D. The advantage of the ResNet algorithm was used to solve the issue of diminishing gradient problems by passing the connection.  Figure 6 shows that in this type of a network, the hidden layers will drop to zero after passing several multiple layers.

## 4. Performance Measure

The following parameters were used to measure the performance of system efficiency: mean, intersection-over-union (IoU), and dice similarity coefficient (DSC).

### 4.1. Mean

The mean reflects the percentage of true positive in each group of pixels as shown in the following equation:

(2) $$\begin{array}{c} \text{Mean}=\frac{T.P}{T.P+T.N}. \end{array}$$

### 4.2. IoU

To identify the difference between the predicted and target output, IoU is applied, which is mentioned in the following equations:

(3) $$\begin{array}{c} \text{Ground truth IOU}=\text{real}\cap \frac{\text{ground truth}}{\text{real}\cup \text{ground truth}}, \end{array}$$

(4) $$\begin{array}{c} \text{IOU value}=\frac{T.P}{T.P+F.P+F.N}. \end{array}$$

### 4.3. D.S.C

The following equation is used to assess the actual and predicted values that are like each other. These values will range from zero to one where one is closer to the actual and predicted value.

(5) $$\begin{array}{c} \text{Predicted value DSC}=2\frac{\text{actual}\cap \text{groundtruth}}{\text{actual}\cup \text{groundtruth}}. \end{array}$$

## 5. Implementation Details

The experiments were run on a server with the windows 10 operating system, 2.30 GHz processor, 128 GB RAM, and NVIDIA Lenovo Think station. The samples were trained by a series of data argumentation, image rotation, zooming, and scaling training samples. The cross-validation process was applied to analyze the proposed model performance.

### 5.1. Database Creation

The freely available datasets were used for experiment purposes. Set 1 and set 2 consist of cropped WBC samples and a set of three raw samples. Jiangxi Tecom Science Corporation, China, provided set 1 containing 300 WBC samples with a size of 120 ∗ 120 and 24 bit color. Set 2 consists of a hundred samples of 300 ∗ 300 size. Set 3 consists of 720 ∗ 576 samples.

### 5.2. Results and Discussion

Figure 7 shows that different intensities are caused due to different illuminations. Hence, the size and shape of the leukocyte vary from each other. The experiment was conducted on the proposed model on publicly available datasets. The six-fold cross-validation was performed on the samples to make sure that all samples were tested properly. The segmentation accuracy of 96% was achieved. The overall comparison of the existing model of various researchers' results was compared with the proposed model as given in Table 2 and the loss function as given in Table 3. The output sample of the proposed sample is shown in Figure 8.

## 6. Conclusion

In this work, the method for identifying and classification of WBC was discussed in detail with the experimental results. The proposed method performed robustness in segmenting WBC, peripheral blood, and bone marrow images with a mean accuracy of 96%. This method can also be applied to the nucleus and cytosol separation. The proposed method can be further continued for better results by using YOLO architecture to identify the objects and classify the same. More object identification and classification techniques can be studied as an extension of this proposed effort to attain better results [32].

## Figures and Tables

**Figure 1:** Sample WBC image [6].

**Figure 2:** Various types of WBCs [6]. (a) Cropped image WBC. (b) Blood smear image. (c) Ground truth image.

**Figure 3:** Classification of white blood cells.

**Figure 4:** Process of segmentation.

**Figure 5:** UNet architecture for WBC.

**Figure 6:** The ResNet architecture model [20].

**Figure 7:** RGB WBC under different illuminations. (a) Image-shade 1. (b) Image-shade 2. (c) Illumination 1st image. (d) Illumination 2nd image.

**Figure 8:** Dataset's samples predicted. (a) Input image. (b) Ground truth image. (c) UNet image. (d) Our model image.

**Table 1:** Layers of the proposed model used.

Layer type	Output	Parameter
I2	(N, 300, 300, 3)	0
EF	(N, 10, 10, 1636)	11783535
Fl	(N, 163500)	0
DP	(N, 163500)	0
DN	(N, 4)	714404
Total params: 12, 497, 939		
Trainable params: 12, 410, 936		
Nontrainable params: 97, 606		

I2, input layer; EF, efficient netblock; Fl, flatten layer; DP, dropout layer; DN, dense layer; N, none.

**Table 2:** Comparison of results sets of existing supervised methods.

Methods of architecture	Mean accuracy	IoU	B.F score	Precision	Recall	Specificity	F1 score
UNet	93.4	90.2	0.65	92.55	97.12	92.74	94.50
SegNet	92.14	85.6	0.52	98.77	97.66	99.89	99.10
FCN	91.34	92.6	0.72	95.65	96.77	97.45	98.67
Proposed method	94.14	95.6	0.92	98.45	97.56	93.23	98.67

**Table 3:** Loss functions of the proposed method.

Dataset	Method	Precision	IoU	FOR	FOR
Set 1, Jiangxi Tekang Technology	*L*=*L*_*B*_CE+*L*_*T*_	95.50	96.2	0.45	1.55
Set 2, Jiangxi Tekang Technology	*L*=*L*_*B*_CE+*L*_*T*_	96.52	97.52	0.35	2.15
Set 3, Jiangxi Tekang Technology	*L*=*L*_*B*_CE+*L*_*T*_	97.52	98.25	0.06	6.05

## Data Availability

The data used to support the findings of this study are available from the corresponding author upon request.
